The article "IL2RB Is a Prognostic Biomarker Associated with Immune Infiltrates in Pan-Cancer" was retracted in 2023. Reasons: signs of a paper mill; suspected computer-generated content; unreliable results or conclusions; concerns about the data.

# IL2RB Is a Prognostic Biomarker Associated with Immune Infiltrates in Pan-Cancer

**DOI:** 10.1155/2022/2043880

**Published:** 2022-04-29

**Authors:** Guangyao Li, Yandong Wang, Ya Cheng

**Affiliations:** ^1^The Second People's Hospital of Wuhu, Department of Gastrointestinal Surgery, East China Normal University, Wuhu 241000, China; ^2^Wuhu Clinical College Affiliated to Nantong University, Wuhu 241000, China; ^3^Department of Emergency Surgery, The First Affiliated Hospital of Anhui Medical University, Hefei 230000, China

## Abstract

**Background:**

Interleukin-2 receptor *β* (IL2RB) is a receptor protein of interleukin-2. IL2RB is implicated in regulation of T cell-mediated immune response. However, the role of IL2RB in pan-cancer is unknown. The present premise sought to explore the role of IL2RB in tumorigenesis, tumor metabolism, and tumor immunity in pan-cancer.

**Methods:**

Data were retrieved from multiple data resources including GTEx data resource, CCLE data resource, TCGA data resource, UCSC data resource, and TISIDB web server. These data were adopted to assess the expression, prognosis value, relationship between IL2RB and immune microenvironment, microsatellite instability, immune new antigen, gene mutation, immune modulatory factors immune checkpoint and TMB, and immune or molecular subtypes of IL2RB in various tumors. Estimate analysis and GSEA were conducted to assess the role of IL2RB in pan-cancer.

**Results:**

Differential analysis illustrated that L2RB was remarkably elevated in pan-cancer, notably in solid tumors compared with normal tissues. Survival analysis indicated that IL2RB was linked to pan-cancer prognosis, and elevated IL2RB contents were remarkably linked to dismal prognosis patients in diverse kinds of cancers. The findings illustrated that IL2RB contents were remarkably linked to tumor immune invasion, tumor microenvironment, TMB, MSI, DNA repair genes, methyl transferases, immune modulatory factors, and immune or molecular subtypes in pan-cancer. IL2RB gene mutation was evident in numerous cancers. The data illustrated that IL2RB contents were remarkably enriched in multiple signaling cascades which modulate tumorigenesis, tumor metabolism along with immunity.

**Conclusion:**

The findings of the present premise illustrate that IL2RB plays an indispensible role in tumorigenesis, tumor metabolism, and immunity. Therefore, it is a prospective target gene in tumor-target therapy and tumor immune therapy. IL2RB is also a valuable predictive biomarker in most solid tumors.

## 1. Introduction

According to the most recent report from the International Agency for Research on Cancer (IARC), about 19.3 million new cases of cancer along with 10.0 million cancer-linked deaths were recorded globally in 2020 [1]. Despite significant progress in diagnosis and treatment of malignant tumor in recent years, most cancer types present poor prognosis. This is mainly attributed to lack of effective diagnostic methods and treatment strategies. Hence, it is pivotal to explore novel biomarkers for diagnosis along with prognosis of cancers to improve cancer management.

The article "IL2RB Is a Prognostic Biomarker Associated with Immune Infiltrates in Pan-Cancer" was retracted in 2023. Reasons: signs of a paper mill; suspected computer-generated content; unreliable results or conclusions; concerns about the data.

Interleukin-2 (IL-2) is a primary immunoregulatory cytokine produced from activated T cells. IL-2 exerts its effects by combining with IL-2R (interleukin-2 receptor) expressed on T cells along with natural killer (NK) cells [2, 3]. IL-2R comprises three subunits: IL-2R*α* (coded by IL2RA), IL-2R*β* (coded by IL2RB), and IL-2R*γ* (coded by IL2RG) [4, 5]. IL2RB gene is a cytokine signaling gene that participates in T cell-triggered immune responses. Studies report that IL2RB is associated with progression of several diseases, for instance, multiple sclerosis, inflammatory bowel disease, and lung cancer [6–8]. However, studies have not fully explored the expression trend and prognostic importance, as well as biological function of IL2RB in cancer. Herein, a comprehensive analysis of IL2RB was conducted to explore the transcription profile, DNA methylation pattern, tumor mutation burden (TMB), mismatch repairs (MMRs), microsatellite instability (MSI) characteristics, association with TME, clinical prognosis value, and role in immune regulation.

## 2. Materials and Methods

### 2.1. Sample Information

Gene expression matrix along with clinical data in tumor and nontumorous samples were retrieved from the GTEx data resource (https://gtexportal.org/), UCSC data resource (https://xenabrowser.net/datapages/), and TCGA data resource (https://portal.gdc.cancer.gov/). Data for 31 cancer samples were obtained from GTEx datasets; data for 5 cancer samples were retrieved from UCSC data resource and 27 cancer samples were obtained from TCGA datasets for analysis in the present study. The CCLE data resource (https://portals.broadinstitute.org/) was utilized to abstract expression data for every tumor cell line. Besides, TIMER data resource (https://cistrome.shinyapps.io/timer/) was employed to abstract pan-cancer immune invasion cell score data. Tumor name acronyms and the match meanings include LUSC (lung squamous cell carcinoma), ACC (adrenocortical carcinoma), WT (high-risk Wilms' tumor), STAD (Stomach adenocarcinoma), BLCA (bladder urothelial carcinoma), CESC (cervical squamous cell carcinoma and endocervical adenocarcinoma), CHOL (cholangiocarcinoma), NB (neuroblastoma), COAD (colon adenocarcinoma), LGG (brain lower grade glioma), COADREAD (colon adenocarcinoma/rectum adenocarcinoma esophageal carcinoma), READ (rectum adenocarcinoma esophageal carcinoma), SARC (sarcoma), BRCA (breast invasive carcinoma), DLBC (lymphoid neoplasm diffuse large B-cell lymphoma), PCPG (pheochromocytoma and paraganglioma), READ (rectum adenocarcinoma), GBM (glioblastoma multiforme), GBMLGG (glioma), MESO (mesothelioma), HNSC (head and neck squamous cell carcinoma), KICH (kidney chromophobe), KIRC (kidney renal clear cell carcinoma), LAML (acute myeloid leukemia), LIHC (liver hepatocellular carcinoma), LUAD (lung adenocarcinoma), OV (ovarian serous cystadenocarcinoma), ESCA (esophageal carcinoma), PAAD (pancreatic adenocarcinoma), PRAD (prostate adenocarcinoma), SKCM (skin cutaneous melanoma), ALL (acute lymphoblastic leukemia), STES (stomach and esophageal carcinoma), TGCT (testicular germ cell tumors), THCA (thyroid carcinoma), THYM (thymoma), UCEC (uterine corpus endometrial carcinoma), UVM (uveal melanoma), OS (osteosarcoma), and KIRC (kidney renal clear cell carcinoma).

The article "IL2RB Is a Prognostic Biomarker Associated with Immune Infiltrates in Pan-Cancer" was retracted in 2023. Reasons: signs of a paper mill; suspected computer-generated content; unreliable results or conclusions; concerns about the data.

### 2.2. Expression Analysis of IL2RB in Pan-Cancer

Differences in IL2RB contents between tumor tissues and nontumorous tissues were evaluated using R software. Difference in the contents of IL2RB between different nontumorous cells and diverse cancer cell lines were explored using Kruskal-Wallis test. Violin plots were constructed via the ggplot R package.

### 2.3. Prognostic Analysis of IL2RB in Pan-Cancer

Univariate survival assessment was performed to explore the association of IL2RB contents with survival of patients. Besides, the Kaplan-Meier approach was utilized to explore the survival rate in pan-cancer with different contents of IL2RB. Tumor along with vicinal non-tumorous tissue samples were categorized into high-IL2RB expression and low-IL2RB expression groups on the basis of the expression levels of IL2RB using the bipartite approach. Univariate Cox survival assessment was performed using survival R package. Data were visualized forest plots.

### 2.4. Association Analysis of IL2RB with the Immune Microenvironment

Tumor-invading lymphocytes are a reliable predictor of sentinel lymph node status as well as cancer survival. Cancer patients' survival is linked to their immune along with stromal scores. Our research method was similar to the former study [9]; the ESTIMATE tool was adopted to explore the relationship of gene expression with immune cell scores. A positive relationship was defined by *P* < .05 coupled with *R* > 0.20.

### 2.5. Association Analysis of IL2RB with Immune Neoantigens along with Immune Checkpoints Genes

A mutated gene in malignant cells codes for neoantigen. The protein is produced as a result of biological events, consisting of point mutations and gene fusions, as well as deletion mutations. The docking affinity score of neoantigen was calculated via antigenic epitopes harboring 8~11 amino acids long. Epitopes harboring a score of less than 500 nm were considered as neoantigens. The predicted neoantigens were ranked according to the docking affinity and variant allele frequency along with antigenicity index values. Using the ScanNeo tool, as similar as research method of former study [9], the number of neoantigens in each tumor sample was measured independently. The link between IL2RB contents with antigen number was also investigated. Moreover, the expression relationship between the top 40 immune checkpoint genes and IL2RB expression was explored. The immune checkpoint genes were abstracted separately, and the correlation between their expression levels and IL2RB expression was determined. *P* < 0.05 and *R* > 0.20 indicated remarkably positive correlations.

The article "IL2RB Is a Prognostic Biomarker Associated with Immune Infiltrates in Pan-Cancer" was retracted in 2023. Reasons: signs of a paper mill; suspected computer-generated content; unreliable results or conclusions; concerns about the data.

### 2.6. Association Analysis of IL2RB with Tumor Mutational Burden and Microsatellite Instability

Tumor mutational burden (TMB) is a measurable marker for quantifying mutations present in a tumor cell. We employed Spearman's rank correlation to assess the TMB of each cancer sample. When comparing tumor tissue to nonmalignant tissue, microsatellite instability (MSI) involves the presence of a novel microsatellite allele. It constitutes any change in the length of a microsatellite produced by the insertion or deletion of a repeat unit. We utilized the Spearman's rank correlation to explore the relationship of IL2RB contents with MSI.

### 2.7. Association Analysis of IL2RB with DNA Mismatch Repair Genes and Methyltransferases

Mismatch repair is a process for repairing mismatches inside cells. When critical genes lose their function as a result of this process, DNA replication mistakes occur that cannot be corrected. These mistakes result in a significant number of somatic mutations. Using expression profile data from the TCGA data resource, the association of five MMR genes (MSH6, MLH1, EPCAM, MSH2, and PMS2) with IL2RB contents was investigated. DNA methylation is a chemical alteration of DNA that affects epigenetic inheritance and modulates gene expression without changing the DNA sequence. The link between IL2RB contents and the expression of four methyltransferases was explored. The ggplot R tool was utilized to visualize the data. The associations were remarkably positive at *P* < 0.05 along with *R* > 0.20.

### 2.8. Gene Set Enrichment Analysis of IL2RB in Pan-Cancer

Gene set enrichment analysis (GSEA) compares genes to predetermined gene sets in order to assess their expression status within a functional gene set. It is also utilized to assess if the expression level is linked to a biological process, a molecular function, or a cellular component [10]. The Kyoto Encyclopedia of Genes and Genomes (KEGG) constitute a comprehensive data resource for genomic, chemical, as well as functional analyses. The Hallmark gene set was employed in GSEA analysis via the molecular signatures database (MsigDB) [11]. The following criteria were used in the GSEA analysis: |NES| >1, *P* < .05, and FDR 0.25. Cascades that satisfied these criteria were deemed to be remarkably enriched [9].

The article "IL2RB Is a Prognostic Biomarker Associated with Immune Infiltrates in Pan-Cancer" was retracted in 2023. Reasons: signs of a paper mill; suspected computer-generated content; unreliable results or conclusions; concerns about the data.

### 2.9. TISIDB Analysis

The TISIDB website comprises 998 immune-linked anticancer genes originated from 4176 records in 2530 studies. The web server is used for analysis of target genes in the tumor immune interplay via analyses of high-throughput data or literature abstraction [12]. Herein, TISIDB was utilized to generate heat maps for exploring the relationship between the contents of IL2RB with immunomodulators and immune cells in diverse kinds of cancer. Further, the relationship of IL2RB contents with immune subtypes or molecular subtypes across human cancers was explored using TISIDB. Besides, the relationship of target genes of some antitumor drugs and *il2rb* gene was evaluated using TISIDB web server. Statistical significance was defined at *P* < .05.

## 3. Results

### 3.1. IL2RB Is Upregulated in Pan-Cancer

The contents of IL2RB in numerous tissues were determined using GTEx data resources, and the expression trend of IL2RB in 31 tissues was described (Figure 1(a)). The expression levels of IL2RB in 21 cell lines were evaluated using data for tumor cell lines retrieved from CCLE data resource (Figure 1(b)). The mRNA contents of IL2RB were abstracted from 20 cancers in TCGA dataset, and a box diagram of the contents of IL2RB in cancers tissues and neighboring tissues was generated (Figure 1(c)). The contents of IL2RB transcript were remarkably higher in KICH, BRCA, STAD, ESCA, GBM, KIRP, HNSC, and KIRC in contrast with the neighboring nontumorous tissues. Data for nontumorous tissues in GTEx data resource and the TCGA malignant tissues were integrated for analysis of the difference in IL2RB contents in 27 tumors (Figure 1(d)). The results demonstrated that the contents of IL2RB were remarkably elevated in 21 tumors tissues relative to nonmalignant tissues.

### 3.2. IL2RB Is a Potential Prognosis Marker in Pan-Cancer

The relationships of the IL2RB mRNA contents with OS (overall survival), DSS (disease-specific survival), DFS (disease-free survival), and PFI (progression-free interval) of 44 cancers were explored. Kaplan-Meier (KM) survival curve coupled with Cox proportional hazards models were utilized to evaluate the prognosis value of IL2RB. The results for Cox regression analyses and correlations between IL2RB with OS, DSS, DFI, and PFI in various cancers were presented as forest plots. The data illustrated that elevated IL2RB contents were not remarkably correlated with DFI (Figure 2(a)). However, IL2RB expression level was negatively associated with DSS in GBMLGG, KIPAN, UVM, LGG, GBM, and KIRP and positively correlated with DSS in SKCM, SKCM-M, THCA, SARC, and HNSC cancer types (Figure 2(b)). Moreover, IL2RB expression level was negatively correlated with OS in GBMLGG, KIPAN, LGG, UVM, GBM, KIRP, THYM, and LAML and positively correlated with OS in SKCM, SACM-M, SARC, and CHOL types (Figure 2(c)). Furthermore, IL2RB expression level was negatively correlated with PFI in GBMLGG, KIPAN, GMB, UVM, LGG, and KIRP cancers and positively correlated with PFI in SKCM, SKCM-M, HNSC, UCEC, and BRCA cancer types (Figure 2(d)).

The article "IL2RB Is a Prognostic Biomarker Associated with Immune Infiltrates in Pan-Cancer" was retracted in 2023. Reasons: signs of a paper mill; suspected computer-generated content; unreliable results or conclusions; concerns about the data.

The results of the KM curve analysis showed that high IL2RB mRNA contents were linked to worse OS in GBM, KIRP, LGG, THYM, and UVM, whereas high IL2RB mRNA levels were associated with better OS in HNSC, SKCM, and SARC (Figure 3(a)). In addition, highIL2RB mRNA levels were correlated with worse DFI in KIRP; worse DSS in GBM, KIRP, LGG, and UVM; and worse PFI in DLBC, KIRP, and LGG. High IL2RB mRNA levels were correlated with better DFI in UCEC, better DSS in SKCM and UCEC, and better PFI in CHOL and UCEC (Figures 3(b)–3(d)).

### 3.3. IL2RB Is Associated with Tumor Immune Invasion and Tumor Microenvironment in Pan-Cancer

Tumor invading lymphocytes are independent prognosis predictors of cancers. The findings in the present work illustrated that IL2RB expression is linked to the level of immune invasion in various cancers, notably in ACC, BRCA, and CHOL (Figure 4). Expression levels of IL2RB were remarkably associated with all six tumor invading lymphocytes including B cells (*R* = 0.463, 0.585, and 0.684, *P* < 0.001), CD4 + T cells (*R* = 0.323, *P* = .0039; *R* = 0.695, *P* < 0.001; and *R* = 0.675, *P* < 0.001), CD8 + T cells (*R* = 0.819, 0.665, and 0.766, *P* < 0.001), dendritic (*R* = 0.614, 0.774, and 0.818, *P* < 0.001), macrophage (*R* = 0.549, 0.293, and 0.759, *P* < 0.001), and neutrophil (*R* = 0.669, 0.742, and 0.496, *P* < 0.001) in ACC, BRCA, and CHOL cancers. Moreover, the stromal score and immune score of individual cancer samples were evaluated via the R package Estimate to explore the roles of IL2RB in tumor immune microenvironment in the course of tumor development. The results showed that the top three tumors with the most remarkable correlation between IL2RB contents and stromal score among the 33 cancers were BLCA (*R* = 0.605, *P* < 0.001), CESC (*R* = 0.426, *P* < 0.001), and ESCA (*R* = 0.541, *P* < 0.001)(Figure 5(a)). BLCA (*R* = 0.605, *P* < 0.001), CESC (*R* = 0.426, *P* < 0.001), and CHOL (*R* = 0.712, *P* < 0.001) were the top three cancers with the most remarkable correlation between IL2RB contents with immune score among 33 cancers (Figure 5(b)). ACC (*R* = 0.598, *P* < 0.001), BLCA (*R* = 0.605, *P* < 0.001), and CESC (*R* = 0.426, *P* < 0.001) were the cancers with the most remarkable correlation between IL2RB contents and estimate immune score (Figure 5(c)).

The article "IL2RB Is a Prognostic Biomarker Associated with Immune Infiltrates in Pan-Cancer" was retracted in 2023. Reasons: signs of a paper mill; suspected computer-generated content; unreliable results or conclusions; concerns about the data.

### 3.4. IL2RB Expression Is Linked to Immune Neoantigens and Immune Checkpoint Genes

To explore the relationship between IL2RB contents with checkpoint gene expression, we combined data from more than forty immune checkpoint genes often detected in diverse kinds of malignancies (Figure 6). The data illustrated that the contents of IL2RB were positively linked with the contents of immune checkpoint genes consisting of THCA, PRAD, and COAD in diverse kinds of malignancies. We established that L2RB modulates the expression of numerous immune checkpoint genes, which plays a pivotal role in modifying tumor immunity. To assess the relationship of IL2RB contents with the amount of these neoantigens, the number of neoantigens in each kind of tumor was evaluated independently. The amount of neoantigens was positively linked with IL2RB contents in LUCA (*R* = 0.24, *P* < .01), UCEC (*R* = 0.189, *P* < .01), CESC (*R* = 0.164, *P* < .05), THCA (*R* = 0.136, *P* < .05), and LGG (*R* = 0.193, *P* < .01) (Figure 7).

### 3.5. IL2RB Expression Is Linked to Tumor Mutational Burden along with Microsatellite Instability in Pan-Cancer

TMB is a measurable marker for quantifying mutations present in malignant cells. TMB constitutes somatic mutation number in the coding sections of a tumor cell genome that occurs at an average of 1 M bases. The total number of nonsynonymous mutations can be easily expressed. Single nucleotide variations (SNVs) along with tiny insertions/deletions constitute the two kinds of mutations that are frequent in many kinds of mutations. Spearman's rank correlation was adopted to assess the relationship of IL2RB contents with TMB in each tumor type. In BLCA, BRCA, COAD, KIRC, LAML, LGG, SARC, THYM, and UCEC, IL2RB contents were positively linked with TMB, whereas in KRIP, PAAD, PRAD, and THCA were inversely linked to TMB (Figure 8).

MSI involves the presence of a novel microsatellite allele in a tumor as compared to neighboring healthy cells as a result of any change in the length of a microsatellite produced by the insertion or deletion of a repeat unit. The relationship of MSI with IL2RB contents was assessed via Spearman's rank correlation. Only COAD was positively linked to IL2RB contents, whereas DLBC, SKCM, ESCA, HNSC, OV, KIRP, MESO, SARC, STAD, LUSC, and TGCT had an inverse relationship with MSI (Figure 9).

The article "IL2RB Is a Prognostic Biomarker Associated with Immune Infiltrates in Pan-Cancer" was retracted in 2023. Reasons: signs of a paper mill; suspected computer-generated content; unreliable results or conclusions; concerns about the data.

### 3.6. IL2RB Affects DNA Mismatch Repair Genes along with Methyltransferase Expression in Pan-Cancer

As illustrated in Figure 10, virtually all of the MMRS genes were positively linked with the contents of IL2RB in about half of the cancers, exhibiting that IL2RB may harbor a role in tumor cell maintenance via upregulation of DNA mismatch repair linked genes. DNA methylation is the covalent coupling of a methyl group to the 5′ carbon position of cytosine in genomic CpG dinucleotides by DNA methyltransferases. We visually explored the association of IL2RB contents with the expression of four methyltransferases and established that IL2RB contents were positively linked to the vast number of cancers, as illustrated in Figure 11. These data illustrated that IL2RB may modulate tumorigenesis along with progression in human pan-cancer via modulating epigenetic status.

### 3.7. IL2RB Modulates Signaling Cascades Involved in Cancer Metabolism along with Tumor Immunity

To assess the influence of gene expression on cancers, human pan-cancer samples were stratified into two groups on the basis of the IL2RB contents: high and low. We utilized GSEA to determine the signaling cascades enriched in the KEGG and HALLMARK data resources in both high and low expression groups. Tables 1 and 2 exhibit the top 20 most enriched signaling cascades or biological processes on the basis of the NES score permutation. We selected the top 3 signaling cascades most enriched in the data resources (Figures 12(a)–12(b)). Cytokine-receptor interaction and complement were the most enriched signaling pathways. These data illustrated that IL2RB plays an indispensable role in modulating signaling cascades participating in tumor immunity along with metabolism.

### 3.8. Relationship between IL2RB and Immune Modulatory Factors in Pan-Cancers

The relationship between IL2RB expression and abundance of tumor-infiltrating lymphocytes (TILs) was explored to determine the role of IL2RB in immune system and its implication in progression of cancers. The data illustrated that IL2RB contents were linked to relative abundance of TILs (such as Act CD8, Tem CD8, and Th1) in most human cancers (Figure 13). Associations between IL2RB expression with immunoinhibitors, immunostimulators, MHCs, chemokines, and receptors were inferred using gene set variation analysis on the basis of the gene expression profile. IL2RB expression levels were positively linked to multiple levels of immunoinhibitors (such as CD96, PDCD1, and TIGIT), immunostimulators (such as CD27, CD28, and CD86), most MHCs (such as HLA-C, HLA-DMA, and HLA-DRA), some chemokines (such as CCL5, CXCL9, and CXCL11), and several receptors (such as CCR1, CCR2, and CXCR6). These data illustrate that IL2RB plays a pivotal role in tumor immunoregulation in Pan-Cancers.

The article "IL2RB Is a Prognostic Biomarker Associated with Immune Infiltrates in Pan-Cancer" was retracted in 2023. Reasons: signs of a paper mill; suspected computer-generated content; unreliable results or conclusions; concerns about the data.

### 3.9. IL2RB Expression Is Associated with Immune and Molecular Subtypes in Pan-Cancers

The TISIDB website was adopted to examine the impact of IL2RB contents on immunological, as well as molecular subtypes in Pan-cancers. C1 (wound healing), C4 (lymphocyte deficient), C2 (IFN-gamma dominant), C5 (immunologically quiet), C3 (inflammatory), and C6 (TGF-b dominant) are the six kinds of immune subtypes. The data exhibiting differential IL2RB expression was among the immune subtypes in various cancers. Expression level of IL2RB was remarkably different among immune subtypes in each cancer type. The top 4 cancer types with the most significant differential IL2RB expression are presented in Figure 14. Further, different molecular subtypes of cancers were remarkably associated with expression of IL2RB.The top 4 tumor types with the most significant differential expression of IL2RB are presented in Figure 15. The results indicate that IL2RB expression differs in immune subtypes and molecular subtypes of diverse human cancers.

### 3.10. IL2RB Is a Target Gene of Several Antitumor Drugs

Data were retrieved from Drug Bank to explore whether IL2RB is a potential target for antitumor drugs. The findings showed that IL2RB gene was a potential target gene for antitumor drugs such as Denileukin diftitox, Aldesleukin, Daclizumab, and Basiliximab (Figure 16 and Table 3). This indicated that IL2RB is a valuable target for antitumor drugs. However, further studies should be conducted to explore the effect of targeting this protein on tumor progression.

## 4. Discussion

Interleukin-2 (IL-2) along with the IL-2 receptor (IL-2R) is the key factor in the regulation of immune system homeostasis and tolerance. IL-2 constitutes a T cell growth factor, which promotes proliferation along with differentiation of activated T cells. IL2RB is part of a receptor signaling complex with pleiotropic functions [13]. IL2RB is activated by endogenous IL2 or therapeutic stimulation, resulting in expression of antitumor immune cell cytokines, such as CD8+ T cells, NK cells, and CD4 + T cells. Previous investigations report that IL2RB is remarkably associated with lung cancer, colorectal cancer, and some autoimmunity diseases [14–16]. However, the role of IL2RB in Pan-cancers has not been fully elucidated.

The article "IL2RB Is a Prognostic Biomarker Associated with Immune Infiltrates in Pan-Cancer" was retracted in 2023. Reasons: signs of a paper mill; suspected computer-generated content; unreliable results or conclusions; concerns about the data.

The findings of the present work exhibited higher contents of IL2RB in pan-cancers, especially in solid tumors in contrast with nontumorous tissues. Moreover, high expression of IL2RB was correlated with worse prognosis in the most tumor types. This indicates that IL2RB plays a key role in tumorigenesis, tumor proliferation, and tumor metastasis.

Tumor invading lymphocytes in TME are independent predictors for cancer prognosis and immunotherapeutic efficacy [17, 18]. Studies report that tumor immune microenvironment is linked to tumorigenesis along with tumor progression [19, 20]. The data herein exhibited that the IL2RB contents were positively linked to the abundance of tumor infiltrating lymphocytes, for instance, CD8 + T cells, dendritic cells, and macrophages in pan-cancers. The expression of IL2RB in ACC, BRCA, and CHOL was positively linked with the abundance of macrophages, which are implicated in immune evasion and suppression [21]. Moreover, more than 40 types of immune-related checkpoint genes including CD274 (PD-L1) were used to further explore the immune-related role of IL2RB. PD-L1 inversely modulates T cell proliferation along with cytokine secretion at a given threshold of T cell receptor attack by binding to PD-1. In addition, it maintains the peripheral tolerance and impairs the immune function of T cell in TME [22, 23]. The findings in the present work indicated that IL2RB expression was remarkably linked to PD-L1 function in most cancer types. Notably, IL2RB was co-expressed with PDCD1 gene, which encodes PD-1 protein. LAG3 is a negative regulator of T cells, and previous findings indicate that blocking LAG3 improves proliferation and activity of cytotoxic T lymphocyte. LAG3 is co-expressed with PD-1 in tumor invading lymphocytes in cancer tissues. Targeting LAG3 combined with PD-1 blockade can alleviate tumor progression and increase regression [24, 25]. The data herein illustrated that IL2RB contents were remarkably linked to LAG3 expression in various cancers. A similar expression trend for IL2RB, PD-1L, and LAG3 in tumors imply that these proteins promote tumor aggressiveness through a common cascade; however, further studies should verify these findings. TMB and MSI remarkably modulate tumor phenotype and patient outcomes [26, 27]. In this premise, IL2RB expression was remarkably linked to TMB or MSI in diverse cancers. However, the effect of IL2RB on TMB or MSI was different in different cancer types. Several investigations are currently exploring tumor immunotherapy to evaluate recovering of antitumor immunoreaction by rebooting and maintaining tumor immune circulation. In the present premise, IL2RB expression was remarkably linked to the expression of key target genes for cancer immunotherapy in pan-cancer. These genes include immunoinhibitors such as CD96 [28, 29], immunostimulators such as CD27 [30], MHCs such as B2M [31], chemokines such as CXCL9 [32], and receptors such as CCR2 [33, 34]. These data illustrate that IL2RB is a potential target gene for development of tumor immunotherapy.

The article "IL2RB Is a Prognostic Biomarker Associated with Immune Infiltrates in Pan-Cancer" was retracted in 2023. Reasons: signs of a paper mill; suspected computer-generated content; unreliable results or conclusions; concerns about the data.

IL2RB is receptor of IL-2, which regulates human immunity by binding IL-2. Studies report that mutations in IL2RB gene reduce surface expression and IL-2 binding, causing T and NK cell-driven immune dysregulation. In addition, high expression of wild-type IL2RB increases IL-2 responsiveness of human T lymphocytes in vitro [35, 36]. Similarly, the results in the current study showed mutation of IL2RB gene in numerous kinds of cancers, implying IL2RB gene plays the role of an oncogene in some cancer types.

Gene set enrichment analysis was performed to explore the role of IL2RB in pan-cancer that was performed for high as well as low IL2RB expression groups. The data illustrated that IL2RB is implicated in several signaling pathways, such as compliment signaling, cytokine-cytokine receptor interaction signaling, PI3K-Akt-mTOR signaling, and allograft-rejection signaling. The highest enrichment scores of these signaling cascades were observed in the high-expression subgroup of IL2RB.This indicates that high IL2RB expression positively modulates these signaling pathways. Moreover, these data illustrate that IL2RB plays a vital role in promoting immune activation, modulating tumor cell viability, and promoting proliferation of tumor cell by upregulating the related signaling cascades.

## 5. Conclusion

In summary, IL2RB expression level is higher in pan-caner tissues relative to the expression level in normal tissues. High IL2RB expression level is associated with worse clinical prognosis in pan-cancers. TMB, MSI, MMRs, and DNA methylation dysregulate IL2RB expression in pan-cancer. In addition, IL2RB is remarkably linked to tumor immune microenvironment and is a potential therapeutic target gene for tumor immunotherapy.

## Figures and Tables

**Figure 1:** IL2RB expression in pan-cancer. (a) Expression levels of IL2RB in a database contain 31 tissues, obtained from the GTEx. (b) Expression levels of IL2RB in a dataset containing 21 tissues in tumor cell lines, collected from the CCLE. (c) Expression levels of ATG5 in tumor and paired adjacent noncancerous tissues containing 20 tissues from TCGA, ∗*P* < 0.05, ∗∗*P* < 0.01, and ∗∗∗*P* < 0.001. (d) IL2RB expression difference in 27 tumors integrating data of normal tissues in GTEx database and data of TCGA tumor tissues, ∗*P* < 0.05, ∗∗*P* < 0.01, and ∗∗∗*P* < 0.001.

The article "IL2RB Is a Prognostic Biomarker Associated with Immune Infiltrates in Pan-Cancer" was retracted in 2023. Reasons: signs of a paper mill; suspected computer-generated content; unreliable results or conclusions; concerns about the data.

**Figure 2:** Forest plot of the relationship between IL2RB expression and DFI (a), DSS (b), OS (c), and PFI (d) time in days, utilizing univariate survival analysis, across 33 types of tumor.

**Figure 3:** The survival curve of IL2RB in pan-cancer using Kaplan-Meier analysis and log-rank test. *P* values<0.05 were considered and shown. (a) The survival curve of IL2RB for OS in 8 kinds of tumor. (b) The survival curve of IL2RB for DFI in 2 kinds of tumor. (c) The survival curve of IL2RB for DSS in 6 kinds of tumor. (d) The survival curve of IL2RB for PFI in 5 kinds of tumor.

**Figure 4:** Analysis for correlation between IL2RB expression in pan-cancer and tumor immune infiltration. (a) Correlation analysis between IL2RB expression and tumor immune infiltration in ACC. (b) Correlation analysis between IL2RB expression and tumor immune infiltration in BRCA. (c) Correlation analysis between IL2RB expression and tumor immune infiltration in CHOL.

**Figure 5:** Analysis for correlation between IL2RB expression in pan-cancer and tumor microenvironment.(a) Correlation analysis between IL2RB expression in pan-cancer and stromal score. (b) Correlation analysis between IL2RB expression in pan-cancer and immune score. (c) Correlation analysis between IL2RB expression in pan-cancer and estimate immune score.

**Figure 6:** Correlation analysis between IL2RB expression and immune checkpoint genes in pan-cancer.

**Figure 7:** Correlation analysis between IL2RB expression and immune neoantigens in pan-cancer.

**Figure 8:** Correlation analysis between IL2RB expression in pan-cancer and TMB.

**Figure 9:** Correlation analysis between IL2RB expression in pan-cancer and MSI.

**Figure 10:** Correlation analysis between the expression of IL2RB in pan-cancer and the expression levels of DNA repair genes.

**Figure 11:** Correlation analysis between the expression of IL2RB in pan-cancer and the expression levels of four types of methyltransferases. DNMT1 is colored red, DNMT2 was colored blue, DNMT3a was colored green, and DNMT3b is colored purple.

**Figure 12:** Gene set enrichment analysis of IL2RB associated with signaling pathways in KEGG and hallmark datasets. (a) Results of GSEA of IL2RB ranked in the top 3 for its association with signaling pathways in KEGG database. (b) Results of GSEA of the top 3 rankings of IL2RB correlation with signaling pathways in hallmark dataset.

**Figure 13:** Immunological correlation between IL2RB and immune modulatory factors in pan-cancers. (a) Spearman correlation between expression of IL2RB and tumor-infiltrating lymphocytes, (b) Spearman correlation between expression of IL2RB and immunoinhibitors, (c) Spearman correlation between expression of IL2RB and immunostimulators, (d) Spearman correlation between expression of IL2RB and MHCs, (e) Spearman correlation between expression of IL2RB and chemokines, and (f) Spearman correlation between expression of IL2RB and receptors across human cancers.

The article "IL2RB Is a Prognostic Biomarker Associated with Immune Infiltrates in Pan-Cancer" was retracted in 2023. Reasons: signs of a paper mill; suspected computer-generated content; unreliable results or conclusions; concerns about the data.

**Figure 14:** The correlation between IL2RB expression and pan-cancer immune subtypes. Note: C1 (wound healing); C2 (IFN-gamma dominant);C3 (inflammatory); C4 (lymphocyte depleted);C5 (immunologically quiet); C6 (TGF-b dominant).

**Figure 15:** The correlation between IL2RB expression and pan-cancer molecular subtypes.

**Figure 16:** 

**Table 1:** The information of KEGG terms from top 20 GSEA enrichment analysis.

Term	ES	NES	NP	FDR	FWER
KEGG_CYTOKINE_CYTOKINE_RECEPTOR_INTERACTION	-0.73989	-2.83535	0	0	0
KEGG_CHEMOKINE_SIGNALING_PATHWAY	-0.74765	-2.83401	0	0	0
KEGG_NATURAL_KILLER_CELL_MEDIATED_CYTOTOXICITY	-0.76894	-2.79488	0	0	0
KEGG_T_CELL_RECEPTOR_SIGNALING_PATHWAY	-0.75892	-2.63393	0	0	0
KEGG_JAK_STAT_SIGNALING_PATHWAY	-0.68386	-2.61912	0	0	0
KEGG_CELL_ADHESION_MOLECULES_CAMS	-0.74518	-2.60315	0	0	0
KEGG_ANTIGEN_PROCESSING_AND_PRESENTATION	-0.80484	-2.5905	0	0	0
KEGG_TOLL_LIKE_RECEPTOR_SIGNALING_PATHWAY	-0.73046	-2.5895	0	0	0
KEGG_HEMATOPOIETIC_CELL_LINEAGE	-0.79373	-2.55457	0	0	0
KEGG_B_CELL_RECEPTOR_SIGNALING_PATHWAY	-0.75321	-2.52634	0	0	0
KEGG_NOD_LIKE_RECEPTOR_SIGNALING_PATHWAY	-0.74814	-2.4982	0	0	0
KEGG_AUTOIMMUNE_THYROID_DISEASE	-0.87166	-2.48917	0	0	0
KEGG_LEISHMANIA_INFECTION	-0.82124	-2.44732	0	0	0
KEGG_TYPE_I_DIABETES_MELLITUS	-0.89289	-2.41995	0	0	0
KEGG_PRION_DISEASES	-0.74146	-2.36926	0	0	0
KEGG_VIRAL_MYOCARDITIS	-0.75558	-2.36393	0	0	0
KEGG_FC_EPSILON_RI_SIGNALING_PATHWAY	-0.63965	-2.33785	0	0	0
KEGG_APOPTOSIS	-0.64052	-2.336	0	0	0
KEGG_LEUKOCYTE_TRANSENDOTHELIAL_MIGRATION	-0.64558	-2.32885	0	0	0
KEGG_FC_GAMMA_R_MEDIATED_PHAGOCYTOSIS	-0.65955	-2.32183	0	0	0

**Table 2:** The information of HALLMARK terms from top 20 GSEA enrichment analysis.

Term	ES	NES	NP	FDR	FWER
HALLMARK_COMPLEMENT	-0.71665	-2.75932	0	0	0
HALLMARK_ALLOGRAFT_REJECTION	-0.83604	-2.74702	0	0	0
HALLMARK_INFLAMMATORY_RESPONSE	-0.75322	-2.65185	0	0	0
HALLMARK_INTERFERON_GAMMA_RESPONSE	-0.83702	-2.60906	0	0	0
HALLMARK_KRAS_SIGNALING_UP	-0.63812	-2.59154	0	0	0
HALLMARK_IL6_JAK_STAT3_SIGNALING	-0.80068	-2.58497	0	0	0
HALLMARK_TNFA_SIGNALING_VIA_NFKB	-0.68369	-2.36623	0	0	0
HALLMARK_INTERFERON_ALPHA_RESPONSE	-0.83745	-2.35777	0	0	0
HALLMARK_APOPTOSIS	-0.57861	-2.26239	0	0	0
HALLMARK_PI3K_AKT_MTOR_SIGNALING	-0.59123	-2.22152	0	1.04E-04	0.001
HALLMARK_APICAL_SURFACE	-0.6112	-2.152	0	8.10E-04	0.006
HALLMARK_APICAL_JUNCTION	-0.55544	-2.09958	0.002037	0.001661	0.011
HALLMARK_EPITHELIAL_MESENCHYMAL_TRANSITION	-0.63205	-1.91513	0.01227	0.009234	0.06
HALLMARK_COAGULATION	-0.48794	-1.79828	0.002058	0.025557	0.156
HALLMARK_MITOTIC_SPINDLE	-0.54658	-1.79733	0.007813	0.024134	0.156
HALLMARK_HYPOXIA	-0.43349	-1.68351	0.029979	0.049823	0.268
HALLMARK_G2M_CHECKPOINT	-0.58366	-1.64297	0.057915	0.060481	0.315
HALLMARK_ANGIOGENESIS	-0.5121	-1.61286	0.048485	0.068585	0.348
HALLMARK_TGF_BETA_SIGNALING	-0.49281	-1.55511	0.067347	0.090498	0.425
HALLMARK_UV_RESPONSE_DN	-0.41845	-1.51394	0.079612	0.106527	0.478

The article "IL2RB Is a Prognostic Biomarker Associated with Immune Infiltrates in Pan-Cancer" was retracted in 2023. Reasons: signs of a paper mill; suspected computer-generated content; unreliable results or conclusions; concerns about the data.

**Table 3:** The relationship between IL2RB gene and target genes of anti-tumor drugs.

ID	Name	Drug type	Targets
DB00004	Denileukin diftitox	Biotech	IL2RA, IL2RB, IL2RG
DB00041	Aldesleukin	Biotech	IL2RA, IL2RB, IL2RG
DB00111	Daclizumab	Biotech	C1QA, C1QB, C1QC, C1R, FCGR1A, FCGR2A, FCGR2B, FCGR2C, FCGR3A, FCG..
DB00074	Basiliximab	Biotech	C1QA, C1QB, C1QC, C1R, C1S, FCGR1A, FCGR2A, FCGR2B, FCGR2C, FCGR3A

## Data Availability

The underlying data supporting the results of our study can be found in GTEx data resource, CCLE data resource, TCGA data resource, UCSC data resource and TISIDB webserver.
